# Effect of Nursing Intervention on Promoting Healing of RW in Patients with Diabetic Foot: A Systematic Review and Meta-Analysis

**DOI:** 10.1155/2022/8284870

**Published:** 2022-10-14

**Authors:** Huan Chen, Xiaoxia Lv, Yingying Zhang

**Affiliations:** ^1^Department of Neurology, Huzhou Central Hospital, Affiliated Central Hospital Huzhou University, Huzhou, 313000 Zhejiang, China; ^2^Orthopedics Department, Huzhou Central Hospital, Affiliated Central Hospital Huzhou University, Huzhou, 313000 Zhejiang, China

## Abstract

**Objective:**

To systematically assess the effect of nursing intervention on promoting the healing of refractory wounds (RW) in patients with diabetic foot (DF).

**Methods:**

A computer search of PubMed, EMBASE, ScienceDirect, CochraneLibrary, China knowledge Network Database (CNKI), China VIP Database, Wanfang Database, and China Biomedical Literature Database (CBM) online database was conducted in a randomized controlled trial (RCT) of traditional Chinese and western medicine nursing intervention on patients with RW of DF. Retrieval time was limited to the period from the date the database was established to present. Separately, two researchers gathered the data. RevMan5.3 statistical software was used to analyze the collected data by meta-analysis according to Cochrane Handbook 5.3.

**Results:**

Finally, 8 articles were included with a total sample size of 772 cases. The meta-analysis of the wound healing time after intervention indicated that the wound healing time of the study group was notably shorter, and the difference was statistically significant (*P* < 0.05). Qualitative, fixed-effect model analysis indicated that the nursing effective rate after treatment in the study group was notably higher, and the difference was statistically significant (*P* < 0.05). Fasting blood glucose level in the study group after treatment was notably lower, and the difference was statistically significant (*P* < 0.05). The life quality in the study group was notably higher, and the difference was statistically significant (*P* < 0.05). Further subgroup analysis indicated that the score of physical function (PF), emotional function (RE), social function (SF), physical pain (BP), general health (GH), vitality (VT), and mental health (MH) in the study group were higher, and the difference was statistically significant (*P* < 0.05). A publication bias analysis was conducted using the inverted funnel chart as the outcome indicator for this study. The results indicated that most of the funnel maps were symmetrical and a few were asymmetrical, suggesting that there exhibited a certain publication bias in the included literature.

**Conclusion:**

The application of traditional Chinese and western medicine nursing intervention when treating DF patients clinically can effectively promote the healing of foot ulcer wounds. Traditional Chinese and western medicine nursing can help patients heal wounds faster and enhance their life quality compared to simplistic western medicine nursing. According to the original literature, the conclusion deserves to be popularized in clinic.

## 1. Introduction

Refractory wounds (RW) are wounds that have failed to heal after more than one month of treatment for various reasons and have no tendency to heal [1]. Diabetes, varicose veins of lower extremities, burns, frostbite, postoperative radiotherapy of cancer, orthopedic postoperative infection, and so on are easy to cause wound nonhealing. Clinical common RW include diabetic foot (DF), traumatic ulcer, compression ulcer, radiation ulcer, venous congestion ulcer, arterial ischemic ulcer, infectious ulcer, and malignant ulcer [2, 3]. DF patients generally have a long course of treatment. This disease is easy to repeat. Long-term failure will lead to excessive consumption, poor nutritional status, decline of physical function, forming a vicious circle, which will not only bring about the decline of the life quality of patients with diabetes, but also cause huge social and economic burden. Wound infections in DF tend to spread to the subcutaneous fat layer and deep tendons. Untimely or improperly treated, the patient's condition can rapidly worsen and eventually lead to amputation, which can be life-threatening in severe cases. Up to now, the use of more advanced molecular biology technology to provide favorable conditions for wound healing, nursing intervention has attached importance to promoting the healing of RW and enhancing the life quality of patients.

The treatment and care of RW such as DF, pressure ulcers, and venous leg ulcers has always been a clinical problem to be overcome. Among various forms of local reflection, foot ulcer is the most common form of manifestation [4]. The clinical features of DF are early extremity numbness, accompanied by pain or no sensation, chills or intermittent claudication, and rest pain [5]. DF refers to patients diagnosed with DM or with a history of DM. Foot infections and severe ulcers can manifest as gangrene, which are often accompanied by diabetic neuropathy or lower extremity vascular disease [6].

Foot ulcers mostly occur 10 years after the onset of diabetes. The longer the course of the disease, the more patients will have neurological disorders of the foot. About 45% of the patients with a course of more than 20 years have neurological disorders of the foot. Recent studies have shown that diabetes people have a 15–40 times higher risk of amputation than nondiabetic patients. Based on the 9th edition of the Global Diabetes Map published by the International Diabetes Federation in 2019, there are currently about 463 million people with diabetes in the world, among which the 20-79-year-old age group, one in every 11 people is a patient. By 2030, 578.4 million people are expected to suffer from DM; by 2045, 700.2 million are expected to suffer from DM [7, 8]. Ninety-two million Chinese people suffer from diabetes today. And there are still 148.2 million adults in the impaired period of glucose regulation, which continues to grow [9]. About 14% of the diabetic patients in China are complicated with DF, among which the risk population of DF is mainly the elderly. One of the vital causes of disability and even death of diabetic patients is DF [10]. 70% of amputations occur in diabetic patients, accounting for more than 50% of all nontraumatic amputations. The mortality rate within 30 days after amputation is about 10%, and the median survival time is 22 months, which is extremely harmful to patients [11].

The clinical value of traditional Chinese and western medicine nursing intervention is explained by the effectiveness of a certain literature or the improvement of a certain evaluation index, which the results are unconvincing. A large number of clinical data have confirmed that integrated traditional Chinese and western medicine nursing has obvious enhancing effect in the healing of ulcer wounds in diabetic group, which has the advantages of less adverse reactions and high patient acceptance [12, 13]. The effect of promoting wound healing in group ulcers has not been internationally recognized and still needs to be supported by high-quality research evidence. In addition, there are large differences between different research designs and many evaluation indicators. There is a great need for more and more authoritative scientific studies to demonstrate the role of Chinese and western nursing interventions in the wound healing of DF ulcers in order to supply a theoretical basis to apply this nursing protocol. Therefore, this study systematically, quantitatively, and comprehensively analyzed the results of multiple independent studies of the same type through meta-analysis.

## 2. Research Contents and Methods

### 2.1. The Sources and Retrieval Methods of Documents

PubMed, EMBASE, ScienceDirect, Cochrane Library, China Journal full-text Database (CNKI), VIP full-text Database (VIP), Wanfang Database, Chinese Biomedical Literature data (CBM), relevant Chinese journals, conference papers, and degree papers were collected. Relevant data was about the nursing effect of traditional Chinese and western medicine nursing intervention on DF patients with difficult wound healing. The literature was searched by the way of free words and subject words, with the key words of nursing intervention, difficult wound healing, traditional Chinese and western medicine nursing, DF, healing effect, meta-analysis, refractory wound, and healing effect from January 2010 to March 2022.

### 2.2. Literature Inclusion Criteria and Exclusion Criteria

The following are the literature inclusion criteria:

1. *Research Type*. All RCT on the effect of nursing intervention of traditional Chinese and western medicine on patients with DF which is difficult to heal
2. *Subjects*. Patients with DF with difficult wound healing were clearly diagnosed. And the diagnostic criteria referred to the relevant diagnostic criteria in the 2010 edition (interpretation of Chinese guidelines to diagnose and treat DF) [14]
3. *Intervention*. The study group received integrated traditional Chinese and western medicine nursing, while the control group only received routine western medicine nursing

The following are the literature exclusion standard:

1. It was not a randomized controlled study
2. There was an incomplete data report, so the data could not be used
3. The content of the study was repeated, and the latest study was taken
4. The assessment of the efficacy of the study was not notable

### 2.3. Quality Evaluation and Data Extraction

1. *Bias Risk Assessment Included in the Study*. For the evaluation, a bias risk assessment tool recommended by Cochrane System Review Manual 5.3 was used
2. *Literature Screening and Data Extraction*. Independently, two researchers screened literature, gathered data, assessed quality, and cross-checked results. When there are differences in opinion, discuss and resolve them or ask the third researcher for help. Research data was managed and extracted using Note Express document management software and Excel office software. A request for additional data would be sent to the author of this article if the data included in the literature were incomplete. The contents of data extraction included (1) basic information as follows: author, publication time, and number of cases; (2) intervention measures as follows: scheme and course of treatment; (3) outcome indicators as follows: nursing effective rate, fasting blood glucose level, wound healing time, and life quality score

### 2.4. Statistical Processing

The standardized mean difference (SMD) with Hedges'*g* was chosen as the measure of the effect. The effect size was calculated using a random-effects model with a restricted maximum-likelihood (REML) and considered a large, moderate, and small effect with respect to the SMD values of 0.8, 0.5, and 0.2, respectively. The heterogeneity among the studies included in a meta-analysis was assessed using Cochrane's *Q*, tau-squared, and *I*-squared (*I*^2^). Cochrane's *Q* test quantifies total variance and generates a *P* value that determines the heterogeneity is present. Tau-squared indicates the true variance that is the between-study variance, while I2 represents the percentage of the total variance that is due to the true variance. The degree of heterogeneity is said to be low, moderate, and high, with I2 values of 25%, 50%, and 75%. RevMan 5.4 software was adopted for meta-analysis. HR and its 95% CI were employed as effect analysis statistics for OS and PFS, and risk ratio and 95% CI were employed as effect analysis statistics for binary variables. *P* and *I*^2^ values in heterogeneity test results were adopted to determine whether there was statistical heterogeneity among the results. *P* > 0.10 and *I*^2^ < 50% indicated that there was no statistical heterogeneity among the research results, and a fixed effect model was used for combined analysis. *P* ≤ 0.10 and *I*^2^ ≥ 50% indicated statistical heterogeneity among the research results, and a random effects model was adopted for combined analysis. The test level of meta-analysis was set as *α* = 0.05. Eggers' test was used to examine the funnel plot asymmetry. Whenever this test was significant with a *P* value of less than 0.1, we used the trim and fill method to correct the funnel plot and adjust the effect size for potential publication bias.

## 3. Results and Analysis

### 3.1. The Results of Literature Retrieval and the Basic Situation of Literature Inclusion

The computer database retrieved 1642 articles, and 528 articles were eliminated when repeated studies were removed. After screening the titles and abstracts of 113 articles, 96 articles were included after eliminating irrelevant studies, reviews, case reports, and no control literature. After carefully reading 88 studies with insufficient data and no major outcome markers, 8 RCTs were eventually included [15–20]. The meta-analysis covered 772 samples in total. All results were shown in Figure 1 and Table 1.

### 3.2. Evaluation of the Quality of the Methodology Included in the Literature

The eight CT articles included in this meta-analysis reported the baseline health status of the patients. All RCT mentioned “random allocation”, of which 6 articles did not describe the randomized method in detail. All gave detailed intervention measures, and only one RCT explained the course of treatment. The number and reasons of blind method and loss of follow-up or withdrawal were not described in detail in 8 RCT articles. According to the Jadad scale, it was found that all the 8 articles had RCT ≤ 2 points (Figures 2 and 3).

### 3.3. Meta-Analysis Result

#### 3.3.1. Wound Healing Time

There were 8 RCTs included in this study with 772 samples. Meta-analysis was conducted on the wound healing time after intervention. The results of the heterogeneity test indicated that Chi^2^ = 60.01, df = 2, *P* < 0.00001 and *I*^2^ = 97%, indicating that the research data contained in the study showed distinct heterogeneity. The random effect model was used to analyze (Figure 4) the wound healing time after intervention, indicated that the wound healing time of the study group was notably shorter than that in control group, and the difference was statistically significant (*P* < 0.05), suggesting that traditional Chinese and western medicine nursing interventions can effectively shorten the healing time of promoting the healing of DF ulcer wounds.

#### 3.3.2. Effective Rate of Nursing

A meta-analysis was conducted on the nursing effectiveness. The results of the heterogeneity test indicated that Chi^2^ = 3.49, df = 4, *P* = 0.48, and *I*^2^ = 0%, indicating that the research data contained in the study showed distinct heterogeneity. The fixed effect model analysis indicated that the nursing effective rate in the study group after treatment was notably higher, and the difference was statistically significant (*P* < 0.05, Figure 5). It suggested the effectiveness of traditional Chinese and western medicine nursing interventions on wound healing of DF ulcers.

#### 3.3.3. Fasting Blood Glucose Level

A meta-analysis of fasting blood glucose levels after intervention indicated that Chi^2^ = 0.01, df = 1, *P* = 0.92, and *I*^2^ = 0%, indicating that the research data contained in the study showed distinct heterogeneity. It can be seen from the fixed effect model analysis (Figure 6), that the level of fasting blood glucose in the study group after treatment was notably lower, and the difference was statistically significant (*P* < 0.05). It suggested that the nursing intervention of traditional Chinese and western medicine could successfully enhance the blood glucose control level of patients with DF.

#### 3.3.4. Life Quality Score

A meta-analysis was conducted on the quality-of-life scores of the patients after intervention. The results of the heterogeneity test indicated that Chi^2^ = 98.07, df = 20, *P* < 0.00001, and *I*^2^ = 80%. The research data contained in the study showed distinct heterogeneity. It could be seen by random effect model analysis (Figure 7) that the life quality of the research group after intervention was notably higher, and the difference was statistically significant (*P* < 0.05). Further subgroup analysis indicated that the scores of PF, RE, SF, BP, GH, VT, and MH in the study group were higher, and the difference was statistically significant (*P* < 0.05).

#### 3.3.5. Publication Bias Analysis

The inverted funnel chart was adopted to measure the publication bias of the study with nursing efficiency as the outcome index (see Figure 8). The results indicated that most of the funnel charts were symmetrical and a few were asymmetrical, suggesting that there was a certain publication bias in the included literature. This may be relevant to the heterogeneity of the study and the small number of included literatures.

## 4. Analysis and Discussion

RW not only seriously affect the life and work of patients, but also an important cause of more serious complications, such as DF has become the primary cause of clinical nontraumatic amputation. Because the mechanism of wound healing is complex and the treatment is difficult, the treatment and nursing of this kind of wound has become a recognized clinical problem. Wound nursing has changed from letting it heal naturally in the past to using bandages, new dressings, creating an environment conducive to wound healing, and nurses' attention to wound exudation, smell, and the progress of wound healing [23]. In recent years, the combination of wound bed theory and wet healing theory has guided a new direction and made a great contribution to the wound treatment of DF. However, the damage to the nerves, blood vessels, muscles, and tendons of the DF caused by high blood sugar, and the changes in the local microenvironment make the wound extremely susceptible to infection and difficult to heal. Even if the wound heals, it is still easy to occur repeatedly [24]. Therefore, patients with DF should go to specialist hospitals for all-round treatment, so as to reduce the disability caused by the continuous deterioration of the disease. At the same time, it is necessary to educate the patients on the knowledge of diabetes and local braking, to change the dressing of the wound regularly in the process of nursing, to avoid friction and weight-bearing, to control the patient's diet, and to take careful care of the patient. It can effectively promote the rehabilitation of patients [25]. This study systematically, quantitatively, and comprehensively analyzed the results of multiple independent studies of the same type through meta-analysis.

Modern medical treatment of DF has a certain effect in controlling blood sugar, improving circulation, nourishing nerve, debridement, and dressing change. Patients have long hospitalization time, long treatment cycle, and high cost, which not only bring great economic pressure to patients but also brings greater burden to society and families. For DF with infection, long-term use of antibiotics will have drug resistance and other problems, which is very difficult. There are also some western medicines when treating digestive tract adverse reactions or other adverse reactions, clinical treatment is faced with many challenges. At the present stage, nursing for patients with DF is the whole treatment process of integrated traditional Chinese and western medicine nursing patients. Flexible application of massage techniques in TCM can greatly reduce the risk of amputation and successfully enhance the survival rate and life quality of patients. According to Chinese medicine, DF belongs to the category of “gangrene”, which is a result of prolonged thirst, resulting in deficiency of both Qi and Yin. If Qi deficiency cannot stimulate the flow of blood, then blood flow is not smooth, meridians are obstructed and limbs cannot be nourished; damp heat is injected and heat toxins accumulate, resulting in pulsatile joint pain and gangrene. Improper treatment and care can lead to aggravation of foot ulcer infection, gangrene and even amputation [26, 27]. Judging from the literature screened and included in this study, a large number of related studies on Chinese and western medicine nursing intervention when treating DF patients have been conducted in China, among which there are many randomized control groups, double-blind, and multicenter high-level studies. It has high clinical application value in patients with DF. There were 8 RCTs included with 772 samples. Qualitative, fixed-effect model analysis indicated that the nursing effective rate after treatment in the study group was notably higher. Traditional Chinese and western medicine nursing interventions are found to enhance the wound healing effect of DF ulcers. The meta-analysis indicated that the nursing intervention of traditional Chinese and western medicine could effectively enhance the blood glucose control level of patients with DF. In the nursing model of traditional Chinese and western medicine, we should pay more attention to the treatment of patients with primary diseases. We can start from the root, take measures such as hypoglycemia and nutritional support to control the blood glucose level of patients with diabetes. The reason why the nursing intervention of traditional Chinese and western medicine can improve the wound healing effect of DF ulcer is that the nursing model can control the blood glucose level of patients through multidimensional nursing intervention, improve local blood circulation and inhibit inflammatory reaction, prevent the occurrence of infection, enhance its body immunity, and then notably improve the effect of ulcer wound healing. The treatment and control of the primary disease are the prerequisites for the treatment of RW. Stabilizing blood sugar, nutritional support, improving blood circulation, nourishing nerves, and enhancing resistance can promote the healing of wounds to a certain extent.

In the aspect of western medicine, psychological nursing, diet nursing, and exercise nursing intervention are the main contents of western medicine nursing work. On the one hand, effective psychological interventions are used to help patients cope with their negative emotions and improve them. The meta-analysis of the wound healing time after intervention indicated wound healing time of the study group was longer. The shortened healing time of ulcer wounds in patients is mainly because the primary disease (diabetes) is controlled. Moreover, targeted measures are taken to inhibit the inflammatory response and nutritional status of the wound, which can effectively enhance the patient's health status and accelerate the recovery of the disease. At the same time, it can effectively control the phenomenon of elevated blood sugar caused by excitement and finally improve the matching degree of patients in the process of treatment. A fair and scientific diet plan can be created by diet nursing taking into account the dietary taboos that patients should be aware of. In addition, exercise nursing can promote the blood circulation of patients and effectively enhance the effect of ulcer healing [28].

In terms of herbal medicine, the absorption of herbs through the patient's acupuncture points by means of foot baths, application, and moxibustion can effectively promote smooth blood circulation. Eliminating the inflammation of the wound to avoid infection of the ulcerated area, thus further promoting the regrowth and development of the tissues and ultimately achieving the therapeutic goal of foot wound healing [29]. In addition, scientific massage on patients' acupoints can effectively stimulate the regulating function of patients themselves through acupoint stimulation, which greatly improve their own immunity and finally effectively promote the speed of wound healing of patients [30]. A meta-analysis was conducted on the quality-of-life scores of the patients after the intervention. The results of the heterogeneity test indicated that the research data contained in the study showed distinct heterogeneity. The random effect model was adopted to analyze the results of the study group. The quality-of-life score was notably higher compared to the control group. It is suggested that the application of traditional Chinese and western medicine nursing in the clinical treatment of diabetic patients can notably enhance the quality of their prognosis. Nursing interventions of integrated traditional Chinese and western medicine are potentially effective to relieve the symptoms of patients. The traditional Chinese medicine nursing techniques are relatively safe and easy to use in prevention and treatment of patients. The main reason why the patient's life quality has been greatly improved is that the disease has been notably relieved. The patient's self-care ability has been notably improved, and the psychological state has also been improved, enabling him to gradually return to normal life. Moreover, nursing interventions have been identified as paramount in managing other relevant chronic conditions, reducing other available risk factors, and establishing physiological condition conducive to greater healing. The monitoring of DF profile, patient activities, and nutritious diet contributes to healing and improves quality of life. Continuous and up-to-date education for nurses caring for patients with DF is another area positively correlated with the efficacy and superiority of the interventions carried out.

Research limitations included that the inclusion and exclusion criteria were relatively strict, and the final number of documents included was relatively small. The result of meta-analysis is not immutable, it is only the result of comprehensive analysis of the existing data. It is considered that with the continuous inclusion and enrichment of new research data, its conclusions should be updated. In the future, it is necessary to conduct more related randomized controlled trials to verify the efficacy. Therefore, it is recommended to carry out more large-sample, multicenter, and high-quality randomized blind studies in strict accordance with the CONSORT statement, to ensure that the follow-up period is long enough and to provide high-quality research evidence for the secondary evaluation with internationally recognized, objective, and transmissible criteria, so as to better evaluate its clinical efficacy, and show the value of promotion.

## 5. Conclusion

To sum up, traditional Chinese and western medicine nursing intervention has a notable effect on enhancing the condition of DF patients with difficult wound healing, which can successfully reduce the blood glucose level of patients, shorten the healing time of DF ulcer wound, and improve their life quality. This intervention method is suitable for clinical application. It is worth popularizing in clinical practice.

## Figures and Tables

**Figure 1:** Illustration of literature screening.

**Figure 2:** Risk bias chart.

**Figure 3:** Summary chart of risk bias.

**Figure 4:** Wound healing time.

**Figure 5:** Nursing efficiency.

**Figure 6:** Fasting blood glucose level.

**Figure 7:** Life quality score.

**Figure 8:** Funnel chart of nursing efficiency.

**Table 1:** Basic characteristics of literature.

Include the literature	Year of publication	N(C/T)	Intervention method		Outcome index	Course of treatment	Stochastic method	Blind or not
			C	T				
Chen [15]	2021	41/41	Routine western medicine nursing	Routine western medicine nursing + TCM nursing	(1)	Unknown	Computer random method	No
Zhong et al. [16]	2018	68/68	Routine western medicine nursing	Routine western medicine nursing + TCM nursing	(1) (4)	6 months	Random number table	No
Luo [17]	2021	45/45	Routine western medicine nursing	Routine western medicine nursing + TCM nursing	(2) (4)	Unknown	Not specified	No
Xiao [18]	2013	35/35	Comprehensive treatment scheme	Comprehensive treatment plus TCM nursing	(1)	Unknown	Not specified	No
Zhong et al. [19]	2019	112/112	Routine western medicine nursing	Routine western medicine nursing + TCM nursing	(1) (3)	Unknown	Not specified	No
Zhong [20]	2019	35/35	Routine nursing intervention	Routine nursing + traditional Chinese and western medicine nursing	(1) (3) (4)	Unknown	Different nursing methods	No
Hu [21]	2016	40/40	Routine western medicine nursing	Routine western medicine nursing + TCM nursing	(1)	Unknown	Not specified	No
Gao and Wang [22]	2019	45/45	Routine western medicine nursing	Routine western medicine nursing + TCM nursing	(2)	Unknown	Not specified	No

Note: C: control group; T: research group. (1) Effective rate of nursing; (2) wound healing time; (3) fasting blood glucose level; (4) life quality score.

## Data Availability

The datasets used and analyzed during the current study are available from the corresponding author upon reasonable request.
